The article "The Effect of Teach-Back Combined with King Interactive Standard Mode on the Life of COPD Patients" was published in 2022. Journal: Contrast Media Mol Imaging.

# The Effect of Teach-Back Combined with King Interactive Standard Mode on the Life of COPD Patients

**DOI:** 10.1155/2022/4638745

**Published:** 2022-09-20

**Authors:** Jiaxi Rang, Liming Peng, Long Wen, Zhiguo Zhou, You Xia, Chaoying Xie, Ting Xie, Jing Tan

**Affiliations:** ^1^Nursing Department, Changsha City First Hospital, Changsha 410000, Hunan, China; ^2^Lao Gan Activity Center, Changsha City First Hospital, Changsha 410000, Hunan, China; ^3^The Department of Respiratory and Critical Care Medicine, Changsha City First Hospital, Changsha 410000, Hunan, China; ^4^Outpatient Office, Changsha City First Hospital, Changsha 410000, Hunan, China

## Abstract

**Background:**

COPD is a common clinical chronic airway inflammatory disease that occurs mostly in middle-aged and older adults over the age of 40. The incidence of COPD is increasing year by year and the onset of age is gradually becoming younger.

**Objective:**

To observe the effect of teach-back combined with king interaction on the life of patients with chronic obstructive pulmonary disease (COPD).

**Methods:**

A total of 100 COPD patients admitted to our hospital from Jan 2021 to Jan 2022 were retrospectively selected to be divided into 50 cases in the control group and 50 cases in the observation group according to the nursing methods. The control group was treated with routine nursing intervention, while the observation group was treated with teach-back combined with king interactive standard mode intervention. The differences in Self-Care Ability Assessment Scale (ESCA) score, St. George's Respiratory Questionnaire (SGRQ) score, Mental State Assessment Scale (MSSNS) score, 6-minute walking distance (6MWD), and pulmonary function indexes were compared between the two groups before and after the intervention. The success rate and patient compliance of each index in the groups were also recorded.

**Results:**

After 3 months and 6 months of intervention, the total SGRO score and its factor scores of self-care skills, self-care responsibility, self-concept, health knowledge level in them were all higher than those before the intervention, while the total SGRO score and its factor scores of respiratory symptoms, activity limitation, disease influence, and so on were all decreased compared with those before the intervention. The ESCA score of the observation group was significantly higher than that of the control one after 3 months and 6 months of intervention, while the SGRQ score was significantly lower than that of the control one, with statistical significance (*P* < 0.05). After 3 months of intervention, the total score of MSSNS and the scores of anxiety, depression, loneliness, and other factors in both groups were decreased compared with those before intervention. After 6 months of intervention, the total score of MSSNS and scores of each factor in both groups were decreased compared with those before intervention, and the MSSNS scores in the observation group were significantly lower than those in the control group after the intervention, which was statistically significant (*P* < 0.05). After 3 months and 6 months of intervention, 6MWD, forced vital capacity (FVC), forced expiratory value in 1 second (FEV1), and FVC/FEV1 in them were all higher than those before intervention, and 6MWD and pulmonary function were significantly higher in the observation group than in the control group after 3 and 6 months of intervention, which was statistically significant (*P* < 0.05). The ESCA score, SGRQ score, MSSNS score, pulmonary function compliance rate, and compliance rate in the observation group were significantly higher than those in the control group, which was statistically significant (*P* < 0.05).

The article "The Effect of Teach-Back Combined with King Interactive Standard Mode on the Life of COPD Patients" was published in 2022. Journal: Contrast Media Mol Imaging.

**Conclusion:**

The use of teach-back combined with king interactive standard mode in COPD patients can improve the patient's self-care ability, reduce psychological negative emotions, and improve the quality of life.

## 1. Introduction

COPD is an airway inflammatory disease characterized by incompletely reversible airflow limitation, with clinical manifestations of chronic cough, sputum, and dyspnea. The symptoms of acute exacerbation are aggravated, and the patients can die from respiratory failure [1, 2]. The main goals of current clinical treatment of COPD are controlling the disease and preventing acute exacerbations. However, the risk of rehospitalization within one year after discharge increases due to the lack of awareness about COPD-related knowledge. The burden of COPD is heavy. It is expected to become the third leading cause of human death by 2030 [3]. Therefore, it is of great importance to improve the self-management ability and life of COPD patients.

Teach-back is a scientific method of communication in which nursing staff provides health education to patients and instructs patients to repeat the knowledge points in their own words to ensure that they really master health knowledge [4]. King interaction standard mode is a mutual pointing interaction model, which deepens the communication and interaction between nurses and patients through the process of perception, judgment, behavior, and response, so as to achieve a good communication effect [5]. The teach-back and king interaction mode have been used in the nursing of respiratory diseases, while the research was not sufficient. In order to improve the awareness rate of COPD-related knowledge and improve the self-management ability of patients and their life quality, the teach-back combined with king interactive compliance model was applied to COPD patients in this study. The report is as follows.

The article "The Effect of Teach-Back Combined with King Interactive Standard Mode on the Life of COPD Patients" was published in 2022. Journal: Contrast Media Mol Imaging.

### 1.1. Core Tips

In this study, the scientific communication model teach-back combined with king interactive compliance model was used to intervene in patients with COPD, and it was found that it could improve the self-care ability of patients, reduce psychological distress, and improve their quality of life.

## 2. Data and Methods

### 2.1. General Information

A total of 100 patients with COPD admitted to our hospital from Jan 2021 to Jan 2022 were retrospectively selected, of whom 59 were males and 41 were females, aged from 40 to 75 years old, with an average of (60.44 ± 8.85) years. The course of disease was 2∼17 years, with an average of (8.96 ± 1.77) years. They were divided into control group (50 cases) and observation group (50 cases) according to the nursing methods. There was no significant difference in specific general data between them (*P* > 0.05).

### 2.2. Case Selection Criteria

Inclusion criteria: (1) in line with the criteria for stable COPD in the Guidelines for the Diagnosis and Treatment of Chronic Obstructive Pulmonary Disease; (2) ages from 18 to 75 years old; (3) having basic verbal communication skills and being able to cooperate with the intervention and assessment of relevant scores; (4) with complete clinical and follow-up data.

Exclusion criteria: (1) with severe mental diseases; (2) presence of in situ or metastatic malignancy; (3) poor overall physical condition with an expected survival of less than six months; (4) inability to perform the 6-minute walk test due to the presence of physical dysfunction; (5) with functional impairment of important organs; (6) long-term bed rest; (7) with hematopoietic system diseases.

### 2.3. Method

In the control group, conventional nursing interventions were used to instruct patients to maintain healthy habits, follow medical prescriptions, perform respiratory function exercises, and pay attention to the prevention of cold, infection, and inhalation of harmful fumes.

The observation group was intervened by teach-back combined with king interactive compliance model. The intervention group of teach-back combined with king interactive compliance model was established, with the nurse manager as the group leader and the charge nurse as the group member. The group was organized to learn COPD rehabilitation training, teach-back and king interactive compliance concept, and other related knowledge. Nursing staff was allowed to join the group after passing the examination. Intervention: (1) Evaluation: One-to-one communication was used on the day of admission or the next day to know the patients' understanding of COPD-related knowledge, self-management ability, willingness, and attitude to participate in interaction. (2) Plan: Develop an intervention plan based on the assessment results by reviewing the relevant literature. The teach-back questionnaire was formulated to carry out the scenario simulation exercise. After that, the existing problems were analyzed and corrective measures were proposed. (3) Implementation: Nursing staff used easy-to-understand language to explain COPD-related knowledge according to the patient's understanding of them, guiding patients to establish a healthy lifestyle, follow medical prescriptions, perform respiratory function exercises, and pay attention to the prevention of cold, infection, and inhalation of harmful fumes. They should ask patients according to the teach-back questionnaire: Did you understand what I just said? What do you agree with? Why is it important to establish a healthy lifestyle, take medication as prescribed, and perform respiratory function exercises? How many times a day do you do respiratory function exercises? How long do you do them each time? Can you show me how to do them? Is there anything else that is unclear to you? If the patient cannot repeat them correctly, the nursing staff should repeat the explanation again. (4) Evaluation: Assess the achievement of the single target value of the plan, analyze the reasons for the failure, and timely adjust the intervention measures. After the patients were discharged from the hospital, the interventions were continued up to 6 months by outpatient follow-up, telephone follow-up or WeChat follow-up, family visits, and other forms.

The article "The Effect of Teach-Back Combined with King Interactive Standard Mode on the Life of COPD Patients" was published in 2022. Journal: Contrast Media Mol Imaging.

### 2.4. Detection Method

Exercise endurance was measured by 6MWD before intervention, 3 months and 6 months after intervention. Patients walked as fast as they could on a flat surface after 15 min of rest, and the walking distance within 6 min was recorded with the unit of meter. The forced vital capacity (FVC) forced expiratory volume in one second (FEV1) with the unit of ml and FVC/FEV1 were measured by German Yager pulmonary function detector.

### 2.5. Score Standard

Self-care ability assessment scale (ESCA) score [6]: evaluation was conducted before intervention, 3 months and 6 months after intervention, including four aspects of self-care skills, sense of responsibility, self-concept, and health knowledge level, with a total of 43 pieces and a single score of 0 to 4. The high ∼ low ESCA score indicates the high ∼ low self-care ability.

Saint George's Respiratory Questionnaire (SGRQ) score [7]: 43 questions were assessed before intervention, 3 and 6 months after intervention, including respiratory symptoms, activity limitation, and disease impact, with 43 questions and a total score range of 0 to 100. The high-low SGRQ score represented the low-high quality of life.

Mental state assessment scale (MSSNS) score [8]: The evaluation was conducted before intervention, 3 months and 6 months after intervention, including four aspects of anxiety, depression, anger, and loneliness, with a total of 38 pieces and a single score of 0 to 4. The high ∼ low MSSNS score indicates the high ∼ low of negative psychology.

Compliance rate: the number of indicators reaching the standard/total number of cases × 100%.

Compliance rate: the self-developed score of this study was used, which covered respiratory function exercise, medication, lifestyle, etc., with a total score range of 0∼100, of which 90 or more points were defined as complete compliance, 60∼89 points as basic compliance, 60 points below as noncompliance. Complete and basic compliance were defined as compliance.

### 2.6. Statistical Method

The data were processed by SPSS26.0. The normality and homogeneity of the measurement data were detected by the K-S method test and Levene's method test, respectively. The measurement data conforming to the standard were described by (*χ* ± *s*). The *t*-test was used for comparison. *χ*^2^ test was applied to compare the count data by the four-compartment table method or the *χ*^2^ test with row × list, and *P* < 0.05 was statistically significant.

## 3. Results

### 3.1. Analysis of Two Groups of General Data

There was no significant difference in the general data of residence, pulmonary function classification, education level, age, gender, and combined diseases between them (*P* > 0.05). See Table 1.

### 3.2. Comparison of ESCA Scores between the Two Groups

Before intervention, there was no significant difference in ESCA score between them (*P* > 0.05). After 3 months and 6 months of intervention, the total SGRO score and its factor scores of self-care skills, self-care responsibility, self-concept, health knowledge level in them were all higher than before, and the ESCA score of the observation group was significantly higher than that of the control one after 3 months and 6 months of intervention, with statistical significance (*P* < 0.05). See Table 2.

### 3.3. Comparison of SGRO Scores between the Two Groups

Before intervention, there was no significant difference in SGRO score between them (*P* > 0.05); the total SGRO score and its factor scores of respiratory symptoms, activity limitation, disease influence, and so on were all decreased compared with those before the intervention, and the SGRO score was significantly lower than that of the control one, with statistical significance (*P* < 0.05). See Table 3.

The article "The Effect of Teach-Back Combined with King Interactive Standard Mode on the Life of COPD Patients" was published in 2022. Journal: Contrast Media Mol Imaging.

### 3.4. Comparison of MSSNS Scores between the Two Groups

Before intervention, there was no significant difference in MSSNS score between them (*P* > 0.05). After 3 months and 6 months of intervention, the total score of MSSNS score and the scores of anxiety, depression, anger (except for 3 months of intervention), and loneliness in them were lower than those before intervention, and the MSSNS score and its factor score (except for anger at 3 months of intervention) in the observation one were significantly lower than those in the control one, with statistical significance (*P* < 0.05). See Table 4.

### 3.5. Comparison of 6MWD and Pulmonary Function between Two Groups

Before intervention, there was no significant difference in 6MWD and pulmonary function indexes between them (*P* > 0.05). After 3 months and 6 months of intervention, the 6MWD, FVC, FEV1, and FVC/FEV1 of them were higher than those before intervention, and the 6MWD and pulmonary function of the observation one were significantly higher than those of the control one after 3 months and 6 months of intervention, with statistical significance (*P* < 0.05). See Figure 1.

### 3.6. Comparison of Two Groups of Indicators Compliance Rate

The ESCA score, SGRQ score, MSSNS score, and lung function compliance rate in the observation one were 90.00% (45/50), 84.00% (42/50), 88.00% (44/50), and 82.00% (82/50), respectively, which were significantly higher than those in the control one with 74.00% (37/50), 66.00% (33/50), 72.00% (36/50), and 64.00% (32/50), respectively, with statistical significance (*P* < 0.05). See Table 5.

### 3.7. Compliance Comparison between Two Groups

The compliance rate of the observation group was 88.00% (44/50), which was significantly higher than 68.00% (34/50) of the control one, with statistical significance (*P* < 0.05). See Table 6.

## 4. Discussion

Dyspnea can not only lead to a decline in exercise endurance and reduce the life quality of patients, but also cause greater economic burden on patients and cause psychological disorders [9, 10]. A survey found that Chinese residents have low awareness of COPD-related knowledge, resulting in about 43% of COPD patients needing hospitalization at least once a year, and more than half of the first-time hospitalized patients died within 3.6 years [11, 12]. Therefore, special attention should be paid to the development and improvement of patients' self-management skills in interventions for COPD to reduce acute COPD exacerbation, which can not only reduce the cost of hospitalization, but also delay the disease and improve the prognosis [13].

The article "The Effect of Teach-Back Combined with King Interactive Standard Mode on the Life of COPD Patients" was published in 2022. Journal: Contrast Media Mol Imaging.

Teach-back method is a simple and practical way of health education, which ensures patients to complete health education better and improve their disease-related knowledge level through explaining, answering, retelling, correcting, and other steps, especially for people with poor health knowledge [4, 14]. At present, teach-back method has been widely used in postoperative rehabilitation, chronic diseases, teaching, and other fields [15, 16]. King interactive standard model believes that the interaction between nurses and patients can help nurses to fully understand the psychological and physiological changes of patients, formulate targeted nursing intervention, and it can stimulate the potential of patients, giving full play to their subjective initiative, which has been applied in obstetrics, surgery, internal medicine, and other fields [17, 18].

In this study, the teach-back combined with king interactive compliance model was applied to the intervention of COPD patients. It was found that the total score of SGRO score and its self-care skills, self-care responsibility, self-concept, health knowledge level of patients after 3 months and 6 months of intervention were higher than those of patients with conventional intervention. The total score of SGRQ score and its respiratory symptoms, activity limitation, and disease impact were lower than those of patients with conventional intervention. Teach-back combined with king interactive compliance model for COPD patients can improve their self-care ability and respiratory function. The results of 6MWD and pulmonary function test suggested that the 6MWD, FVC, FEV1, and FVC/FEV1 of the intervention group using teach-back combined with king interactive compliance model after 3 and 6 months of intervention were higher than those of the conventional intervention one, and the ESCA score, SGRQ score, MSSNS score, and pulmonary function compliance rate were significantly higher than those of the conventional intervention one. The results suggested that teach-back combined with king interactive compliance model for COPD patients could improve exercise tolerance and pulmonary ventilation function, which was due to the fact that the teach-back method eliminated the one-way information transmission mode of routine health education and evaluated and provided feedback on patients' knowledge mastery through retelling to help patients better grasp and understand health education information [19, 20]. In the process of king interactive standard intervention, it focuses on the interaction between nurses and patients and strengthens health knowledge through the spiral process of continuous cognition, error correction, and recognition, so as to improve the self-management ability of patients, stimulate their subjective initiative, and better implement the compliance behavior [21–23]. In the king interactive compliance model, nurses participate in the whole process of interaction, which can discover the problems in the plan and adjust the intervention scheme in time to ensure the continuity of intervention [24, 25].

The article "The Effect of Teach-Back Combined with King Interactive Standard Mode on the Life of COPD Patients" was published in 2022. Journal: Contrast Media Mol Imaging.

COPD patients have decreased motor function due to somatic symptoms, and some patients even lose their ability to work and self-care in daily life, which causes negative emotions [26–28]. Severe negative emotion can affect patients' sleep quality and their treatment compliance, which is detrimental to the prognosis [29–31]. The study found that the total MSSNS score and its factor scores at 3 months and 6 months of the teach-back combined with king interactive compliance model were lower than those who used the conventional intervention, and the compliance rate was higher than that of the conventional intervention. It suggests that teach-back combined with king interactive compliance model for COPD patients can reduce the negative emotions of patients and improve treatment compliance. This is due to the fact that patients in teach-back combined with king interactive compliance model have better mastery of disease-related knowledge and pay more attention to disease treatment and compliance behavior, resulting in an increased compliance. Patients communicate with nursing staff throughout the process in this model, so as to find out their negative emotions and get timely relief, thus reducing their negative emotions [32, 33].

There were some limitations of this study. This study was a retrospective study, and the selection bias was inevitable. Furthermore, the sample of this study was only 100 patients. And finally, this study was performed in only one hospital. Thus, the results should be confirmed by further multicenter randomized controlled clinical trials.

In conclusion, teach-back combined with king interactive compliance model for COPD patients can improve their self-care ability, reduce psychological distress, and improve the quality of life.

## Figures and Tables

**Figure 1:** The FVC, FEV1, FVD/FEV1, and 6MWD of two groups before intervention, 3 months after intervention and 6 months after intervention.

**Table 1:** Analysis of the general data of the two groups.

Normal information	Control one (*n* = 50)	Observation one (*n* = 50)	*χ* ^2^ or *t*	*P*
Gender [*n*(%)]			1.034	0.309
Male	27 (54.00)	32 (64.00)		
Female	23 (46.00)	18 (36.00)		
Age [$\left(\bar{\chi }\pm s\right)$, age]	61.42 ± 9.43	59.86 ± 10.04	0.801	0.425
Body mass index [$\left(\bar{\chi }\pm s\right)$, kg/m^2^]	24.51 ± 2.12	24.39 ± 2.25	0.274	0.784
Course of disease [$\left(\bar{\chi }\pm s\right)$, year]	8.67 ± 1.85	9.05 ± 1.77	1.049	0.297

Place of residence [*n*(%)]			0.161	0.688
City	28 (56.00)	26 (52.00)		
Rural	22 (44.00)	24 (48.00)		

Pulmonary function class [*n*(%)]			0.486	0.784
Class I	28 (56.00)	25 (50.00)		
Class II	16 (32.00)	17 (34.00)		
Class III	6 (12.00)	8 (16.00)		

Educational level [*n*(%)]			0.963	0.618
Junior high school and below	18 (36.00)	15 (30.00)		
High school and secondary school	22 (44.00)	21 (42.00)		
College and above	10 (20.00)	14 (28.00)		

Concomitant disease [*n*(%)]				
Hypertension	17 (34.00)	14 (28.00)	0.421	0.517
Diabetes	8 (16.00)	12 (24.00)	1.000	0.317
Cerebrovascular disease	14 (28.00)	15 (30.00)	0.049	0.826
Hyperlipidemia	9 (18.00)	11 (22.00)	0.250	0.617

The article "The Effect of Teach-Back Combined with King Interactive Standard Mode on the Life of COPD Patients" was published in 2022. Journal: Contrast Media Mol Imaging.

**Table 2:** Comparison of ESCA scores between the two groups [(*χ* ± *s*), fraction].

Factor	Time	Control one	Observation one	*t*	*P*
		*n* = 50	*n* = 50		
Self-care skills	Before intervention	20.55 ± 4.78	20.46 ± 4.83	0.094	0.926
	Intervention for 3 months	26.88 ± 5.11^*∗*^	30.13 ± 5.15^*∗*^	3.168	0.002
	Intervention for 6 months	32.25 ± 6.62^*∗*^	39.25 ± 7.14^*∗*^	5.084	<0.001

Self-care responsibility	Before intervention	14.25 ± 3.28	14.09 ± 3.31	0.243	0.809
	Intervention for 3 months	16.88 ± 3.33^*∗*^	18.96 ± 3.29^*∗*^	3.142	0.002
	Intervention for 6 months	19.54 ± 3.17^*∗*^	22.45 ± 3.69^*∗*^	4.230	<0.001

Self-concept	Before intervention	17.44 ± 3.13	17.52 ± 2.97	0.131	0.896
	Intervention for 3 months	19.05 ± 3.05^*∗*^	21.53 ± 3.39^*∗*^	3.846	<0.001
	Intervention for 6 months	22.96 ± 3.45^*∗*^	25.85 ± 3.59^*∗*^	4.104	<0.001

Health knowledge level	Before intervention	41.08 ± 8.22	40.73 ± 8.69	0.207	0.837
	Intervention for 3 months	45.45 ± 6.78^*∗*^	49.63 ± 8.85^*∗*^	2.900	0.005
	Intervention for 6 months	50.22 ± 7.89^*∗*^	57.14 ± 7.61^*∗*^	4.464	<0.001

ESCA total score	Before intervention	93.32 ± 9.04	92.87 ± 10.11	0.235	0.815
	Intervention for 3 months	108.26 ± 12.78^*∗*^	120.25 ± 13.69^*∗*^	4.527	<0.001
	Intervention for 6 months	124.97 ± 15.47^*∗*^	144.69 ± 18.55^*∗*^	5.773	<0.001

^*∗*^ *P* < 0.05 indicates the comparison with the control group.

**Table 3:** Comparison of SGRQ scores between the two groups [(*χ* ± *s*), fraction].

Factor	Time	Control one	Observation one	*t*	*P*
		*n* = 50	*n* = 50		
Respiratory symptoms	Before intervention	63.25 ± 6.85	64.32 ± 6.72	0.788	0.432
	Intervention for 3 months	53.77 ± 5.16^*∗*^	49.08 ± 5.46^*∗*^	4.414	<0.001
	Intervention for 6 months	46.26 ± 5.58^*∗*^	43.56 ± 5.05^*∗*^	2.537	0.013

Limited activity	Before intervention	60.74 ± 7.88	59.65 ± 7.96	0.688	0.493
	Intervention for 3 months	52.77 ± 7.45^*∗*^	46.32 ± 6.39^*∗*^	4.647	<0.001
	Intervention for 6 months	45.36 ± 5.97^*∗*^	40.45 ± 4.82^*∗*^	4.525	<0.001

Disease impact	Before intervention	61.78 ± 7.12	62.67 ± 6.31	0.661	0.510
	Intervention for 3 months	54.55 ± 6.85^*∗*^	49.44 ± 6.66^*∗*^	3.782	<0.001
	Intervention for 6 months	44.89 ± 5.34^*∗*^	41.28 ± 5.13^*∗*^	3.447	0.001

Overall SGRQ score	Before intervention	61.92 ± 5.88	62.21 ± 6.03	0.243	0.808
	Intervention for 3 months	53.69 ± 5.41^*∗*^	48.28 ± 5.11^*∗*^	5.140	<0.001
	Intervention for 6 months	45.50 ± 4.97^*∗*^	41.76 ± 4.57^*∗*^	3.917	<0.001

^*∗*^ *P* < 0.05 indicates the comparison with the control group.

The article "The Effect of Teach-Back Combined with King Interactive Standard Mode on the Life of COPD Patients" was published in 2022. Journal: Contrast Media Mol Imaging.

**Table 4:** Comparison of MSSNS scores between the two groups [(*χ* ± *s*), fraction].

Factor	Time	Control one	Observation one	*t*	*P*
		*n* = 50	*n* = 50		
Anxiety	Before intervention	24.21 ± 3.77	24.08 ± 4.56	0.155	0.877
	Intervention for 3 months	22.74 ± 3.12^*∗*^	21.51 ± 2.98^*∗*^	2.016	0.047
	Intervention for 6 months	20.39 ± 2.63^*∗*^	19.23 ± 3.12^*∗*^	2.010	0.047

Depression	Before intervention	15.88 ± 2.12	15.79 ± 2.26	0.205	0.838
	Intervention for 3 months	13.73 ± 2.05^*∗*^	12.26 ± 1.79^*∗*^	3.819	<0.001
	Intervention for 6 months	11.64 ± 1.85^*∗*^	10.25 ± 1.74^*∗*^	3.870	<0.001

Anger	Before intervention	10.56 ± 2.44	10.48 ± 2.36	0.167	0.868
	Intervention for 3 months	9.87 ± 2.11	9.71 ± 1.98	0.391	<0.001
	Intervention for 6 months	9.46 ± 1.89^*∗*^	8.34 ± 1.45^*∗*^	3.325	0.001

Lonely	Before intervention	13.66 ± 2.54	13.74 ± 2.48	0.159	0.874
	Intervention for 3 months	12.06 ± 2.13^*∗*^	10.58 ± 1.91^*∗*^	3.658	<0.001
	Intervention for 6 months	9.65 ± 1.82^*∗*^	8.77 ± 1.65^*∗*^	2.533	0.013

MSSNS total score	Before intervention	64.31 ± 5.22	64.09 ± 4.93	0.217	0.829
	Intervention for 3 months	58.41 ± 4.53^*∗*^	54.06 ± 4.11^*∗*^	5.029	<0.001
	Intervention for 6 months	51.14 ± 4.15^*∗*^	48.87 ± 4.03^*∗*^	2.775	0.007

^*∗*^ *P* < 0.05 indicates the comparison with the control group.

**Table 5:** Comparison of the compliance rate of each index between the two groups [*n*(%)].

Group	*n*	ESCA score compliance rate	SGRQ score compliance rate	MSSNS score compliance rate	Pulmonary function compliance rate
Control one	50	37 (74.00)	33 (66.00)	36 (72.00)	32 (64.00)
Observation one	50	45 (90.00)	42 (84.00)	44 (88.00)	41 (82.00)
*χ* ^2^		4.336	4.320	4.000	4.110
*P*		0.037	0.038	0.046	0.043

**Table 6:** Comparison of compliance between the two groups [*n*(%)].

Group	*n*	Full compliance	Basic compliance	Noncompliance	Compliance rate
Control one	50	14 (28.00)	20 (40.00)	16 (32.00)	34 (68.00)
Observation one	50	32 (64.00)	12 (24.00)	6 (12.00)	44 (88.00)
*χ* ^2^					5.828
*P*					0.016

The article "The Effect of Teach-Back Combined with King Interactive Standard Mode on the Life of COPD Patients" was published in 2022. Journal: Contrast Media Mol Imaging.

## Data Availability

The datasets used and analyzed during the current study can be obtained from the corresponding author upon reasonable request.
